# Contrastive study of two screening criteria for active surveillance in patients with low-risk papillary thyroid microcarcinoma: a retrospective analysis of 1001 patients

**DOI:** 10.18632/oncotarget.19503

**Published:** 2017-07-22

**Authors:** Kai Qian, Kai Guo, Xiaoke Zheng, Tuanqi Sun, Duanshu Li, Yi Wu, Qinghai Ji, Zhuoying Wang

**Affiliations:** ^1^ Department of Head and Neck Surgery, Fudan University Shanghai Cancer Center, Shanghai 200032, China; ^2^ Department of Oncology, Fudan University Shanghai Medical College, Shanghai 200032, China

**Keywords:** screening criteria, active surveillance, papillary thyroid microcarcinoma, prognostic indicators, retrospective study

## Abstract

Screening out patients who do not require immediate surgery is a growing trend in the field of thyroid research. In this study, we retrospectively compared the application of two surveillance selection criteria in 1001 patients who had undergone surgical treatment of papillary thyroid microcarcinoma (PTMC): low-risk PTMC characteristics defined by Kuma Hospital and CATO consensus on PTMC management of active surveillance. Treatment outcomes were compared between groups. We then analyzed the prognostic indicators of patients who could be managed by surveillance. A total of 724 patients met Kuma screening criteria and 135 met CATO screening criteria. The Kuma low-risk group had a lower incidence of multifocal lesions and CLNM than Kuma high-risk group. We also found more obvious differences in multifocal lesions, CLNM and extrathyroidal extension when evaluating the CATO low-risk criteria in the same manner. On the other hand, patients in the CATO low-risk group had a lower disease progression rate and longer disease-free survival than those in CATO high-risk group. There was no significant difference in prognosis between the Kuma low-risk group and Kuma high-risk group. Our logistic regression analysis showed that a preoperative ultrasound size of >5 mm, male sex, younger age, and malignant lesions without concurrent benign nodules could be predictors of CLNM. In conclusion, patients classified in CATO low-risk criteria had lower proportion of clinicopathological risk factors than the ones in Kuma low-risk criteria. We also found more risk factors may not be suitable for surveillance, such as tumors without concurrent benign nodules.

## INTRODUCTION

Papillary thyroid microcarcinoma (PTMC) is defined as papillary thyroid cancer (PTC) of ≤10 mm regardless of the existence of distant metastasis [1]. Based on epidemiological studies of different countries, the incidence of thyroid cancer has continuously increased as shown by the widespread use of ultrasonography and fine-needle aspiration (FNA) technology during the past few decades [2–4]. The greatest contribution to this increase in thyroid cancer is the increase in PTMC [5]. The characteristics of PTMC, such as its low distant metastasis rate, high survivability, and inevitable incision scars and surgical complications have caused surgeons to suspect that surgical treatment is necessary for patients with PTMC. However, is small-volume PTC equivalent to low-risk lesions? The answer is clearly no. We identified a non-negligible proportion of patients with PTMC who had cervical lymph node metastasis and other risk factors likely to promote progression of the disease if not surgically treated [6,7].

Therefore, how to distinguish between harmless and harmful PTMC and improve patients’ quality of lives is the main clinical question. A variety of methods have been used in an attempt to address this issue, including thyroid lobectomy alone for low-risk PTMC [8] and new technologies that reduce surgery-related negative effects. Notably, some scholars have attempted to establish several screening criteria with which to select patients with harmless PTMC suitable for management by surveillance rather than immediate surgery. In their analysis of the treatment of low-risk PTC, Brito *et al.* [9] also proposed that active surveillance is especially appropriate for some patients with PTC considering the cost, complications, and prognosis. These authors later established a detailed risk stratification for use when considering active surveillance as an alternative to immediate surgery in patients with PTMC with the goal of helping clinicians to determine the appropriateness of an observational management approach [10]. To prove the feasibility of active surveillance for low-risk PTMC and identify the characteristics of harmless lesions, we performed a retrospective study in which two such criteria were applied to our patients who had undergone surgical treatment: low-risk PTMC characteristics defined by Kuma Hospital and Chinese Association of Thyroid Oncology (CATO) consensus on PTMC management by active surveillance [11,12]. The aim of this study was to obtain authentic clinicopathological characteristics and identify the main indications for strict active surveillance.

## RESULTS

### Patient characteristics

From 2007 to 2010, a total of 3121 patients diagnosed with PTC underwent surgical treatment at our hospital. Of these patients, 1243 (39.8%) patients accepted operations for consideration of PTMC and were proved histologically. Finally, 1001 patients with PTMC who met the study conditions were included (Figure 1). Of these 1001 patients, 724(72.3%) met the Kuma screening criteria and 135 (13.5%) met the CATO screening criteria. The patients comprised 228 male and 773 female patients ranging in age from 16 to 77 years. A total of 106 patients underwent total thyroidectomy while the other 895 patients underwent lobectomy with or without subtotal resection of the contralateral lobe. Recurrence or metastasis was found in 57 patients during follow-up (contralateral lobe recurrence, n = 34; cervical lymph node recurrence, n = 14; both contralateral lobe and lymph node recurrence, n = 6; lung metastasis, n = 2; and contralateral lobe recurrence with sternum metastasis, n = 1). Four patients died of causes unrelated to their thyroid neoplasm (Table 1).

**Figure 1:** 2007-2010 PTC patients undergoing operations in our hospital

**Table 1:** Clinical pathological characteristics of 1001 PTMC patients

	Clinicopathological characteristics	No.
Preoperative information	Age (year)	
	Mean±SD	45.28±10.09
	≤45/>45	524(52.3)/447(44.7)
	Male/female	228(22.7)/773(77.2)
	Familial history	41(4.1)
	Radiation exposure	9(0.9)
	Hashimoto thyroiditis	236(23.6)
	Size by ultrasound (mm)	7.57±1.87
	LNM in preoperative examination	146(14.6)
	Multifocal lesions	98(9.8)
	MT concurrent with benign nodules	531(53.0)
Intraoperative information	Surgical approach	
	Thyroid lobectomy	895(89.4)
	Near-total or total thyroidectomy	106(10.6)
	Subtype	
	Ordinary	984(98.3)
	Follicular variant	15(1.5)
	Oncocytic variant	2(0.2)
	Multifocal lesions	167(16.7)
	Extrathyroidal extensions	75(7.5)
	Neck dissection	
	CLNM	362(36.2)
	LLNM	86(8.6)
Postoperative information	Recurrence and metastasis	57(5.7)
	Death	4(0.4)
	Follow-up time(month)	77.16±18.80
	Temporary hypoparathyroidism	34(3.4)
	Temporary vocal cord paralysis	36(3.6)
	Permanent vocal cord paralysis	24(2.4)

Data were presented as n (%) or mean± standard deviation.

CLNM, central lymph node metastasis.

LLNM, lateral lymph node metastasis.

### Comparisons of characteristics among groups

According to the grouping definition, comparisons were made between the Kuma low- and high-risk PTMC groups and between the CATO low- and high-risk PTMC groups. Patients in the Kuma low-risk PTMC group had a significantly lower incidence of some potentially dangerous characteristics than patients in the Kuma high-risk PTMC group, such as multifocal lesions (14.8% vs. 21.7%, respectively; p < 0.05) and central lymph node metastasis (CLNM) (30.9% vs. 49.8%, respectively; p < 0.05), but not external invasion (6.5% vs. 10.1%, respectively; p = 0.060). We also found obvious differences in all pathological characteristics (multifocal lesions, external invasions, and CLNM) between the CATO low- and high-risk PTMC groups. The results of these comparisons were shown in Table 2. Evaluation of surgical complications showed that the ratio of adverse events remained low in all surgery patients and that no significant differences were present between the groups (data not shown).

**Table 2:** Comparative analysis of patients in different groups

Pathologic characteristics and prognostic factors	Groups		P value	Groups		P value
	Kuma low-risk group	Kuma high-risk group		CATO low-risk group	CATO high-risk group	
**Multifocal lesions**			**0.011**			**0.000**
Positive	107(14.8)	60(21.7)		9(6.7)	158(18.2)	
Negative	617(85.2)	217(78.3)		126(93.3)	708(81.8)	
**Extrathyroidal extensions**			0.060			**0.008**
Positive	47(6.5)	28(10.1)		3(2.2)	72(8.3)	
Negative	677(93.5)	249(89.9)		132(97.8)	794(91.7)	
**CLNM**			**0.000**			**0.000**
Positive	224(30.9)	138(49.8)		25(18.5)	337(38.9)	
Negative	500(69.1)	139(50.2)		110(81.5)	529(61.1)	
**Recurrence/metastasis**			0.127			**0.025**
Positive	36(5.0)	21(7.6)		2(1.5)	55(6.4)	
Negative	688(95.0)	256(92.4)		133(98.5)	811(93.6)	

Data were presented as n (%).

Group comparisons of factors were using the Chi-square test or Fisher's exact probabilities test.

Table 2 and Figure 2 also show the differences in disease progression in patients who satisfied the two criteria. Thirty-six of the 57 patients who experienced recurrence or distant metastasis satisfied the Kuma Hospital screening criteria, while only 2 patients satisfied the CATO screening criteria. Patients in the CATO low-risk PTMC group had a lower progression rate than those in the CATO high-risk PTMC group (1.5% vs. 6.4%, respectively; p < 0.05). This difference in the progression rate was not statistically significant when applying the Kuma low-risk criteria to the comparison, although the ratio was lower in the low-risk PTMC group (5.0% vs. 7.6%, respectively; p = 0.127). Using the Kaplan–Meier method, we also found that the CATO low-risk PTMC group had significantly longer disease-free survival (DFS) than the CATO high-risk PTMC group, while there was no significant difference in DFS between the Kuma low- and high-risk PTMC groups (Figure 2A and 2B).

**Figure 2:** Kaplan-Meier analyses of disease-free survival (DFS) of patients in different groups (Log-rank tests **(A)**: χ2=2.953, P=0.086. **(B)**: χ2=5.324, P=0.021. **(C)**: χ2=4.433, P=0.035.)

Based on the above data, the CATO low-risk criteria seemed to show more pronounced effects in distinguishing the harmless lesions. Because the CATO low-risk PTMC group was contained within the Kuma low-risk PTMC group, we attempted further comparison by dividing the Kuma low-risk patients into two groups that would directly reflect the differences between the two criteria. The patients in the CATO low-risk PTMC group showed a lower incidence of multifocal lesions (6.7% vs. 16.6%, p < 0.05), extrathyroidal extensions (2.2% vs. 7.5%, p < 0.05), CLNM (18.5% vs. 33.8%, p < 0.05), progression rates (1.5% vs. 5.8%, p < 0.05), and prolonged DFS (Table 3, Figure 2C).

**Table 3:** Comparative analysis of low-risk patients in different groups

Pathologic characteristics and prognostic factors	Groups		P value
	CATO low-risk group	Kuma-CATO group	
**Multifocal lesions**			**0.003**
Positive	9(6.7)	98(16.6)	
Negative	126(93.3)	491(83.4)	
**Extrathyroidal extensions**			**0.031**
Positive	3(2.2)	44(7.5)	
Negative	132(97.8)	545(92.5)	
**CLNM**			**0.000**
Positive	25(18.5)	199(33.8)	
Negative	110(81.5)	390(66.2)	
**Recurrence/metastaisis**			**0.045**
Positive	2(1.5)	34(5.8)	
Negative	133(98.5)	555(94.2)	

Data were presented as n (%).

Group comparisons of factors were using the chi-square test or Fisher's exact probabilities test.

Kuma-CATO group presented the 589 patients satisfied the Kuma Hospital screening criteria but not the CATO screening criteria.

### Independent predictors of CLNM and DFS

The independent predictors of CLNM were analyzed using logistic regression, and a Cox proportional hazards regression model was used to assess the risk factors for DFS. When analyzing independent predictors of CLNM in patients with low-risk PTMC, we only considered demographic data and preoperative examination findings because the postoperative pathology was unavailable for management by active surveillance. The multivariate logistic regression analyses showed male sex, younger age, preoperative ultrasound size of >5 mm, and malignant lesions not concurrent with benign nodules were significantly associated with CLNM (Table 4). Familial history, radiation exposure, and Hashimoto thyroiditis were not statistically significant predictors of CLNM.

**Table 4:** Univariate and multivariate logistic regression for CLNM in low-risk PTMC patients

Variables	Univariate		Multivariate	
	OR (95% CI)	P value	OR (95% CI)	P value
Gender (female vs.male)	1.781(1.238-2.563)	**0.002**	1.614(1.105-2.357)	**0.013**
Age (>45 vs.≤45 yr)	1.667(1.212-2.293)	**0.002**	1.548(1.113-2.153)	**0.009**
Familial history	1.433(0.683-3.005)	0.341		
Hashimoto thyroiditis	0.923(0.625-1.364)	0.689		
Radiation exposure	4.573(0.412-50.773)	0.216		
Size by ultrasound (≤5 vs. >5 mm)	2.106(1.338-3.316)	**0.001**	1.931(1.217-3.066)	**0.005**
Multifocal lesions in preoperative examination	1.987(1.150-3.433)	**0.014**	1.592(0.902-2.811)	0.109
MT concurrent with benign nodules (+ vs -)	1.951(1.418-2.684)	**0.000**	1.661(1.193-2.314)	**0.003**

OR, odds ratio; CI, confidence interval.

In the univariate analysis of the predictors of DFS, the significant risk factors were radiation exposure, preoperative ultrasound size of >5 mm, and malignant lesions not concurrent with benign nodules (log-rank analysis). However, the Cox proportional hazards regression model showed that the only risk factor was malignant lesions not concurrent with benign nodules (Table 5).

**Table 5:** Univariate and multivariate analysis for disease-free survival in low-risk PTMC patients

Variables	Univariate	Multivariate	
	P value	HR (95% CI)	P value
Gender (female vs. male)	0.682		
Age (>45 vs.≤45 yr)	0.298		
Familial history	0.203		
Hashimoto thyroiditis	0.147		
Radiation exposure	**0.025**	6.702(0.912-49.234)	0.062
Size by ultrasound (≤5 vs. >5 mm)	**0.030**	3.880(0.930-16.192)	0.063
Multifocal lesions in preoperative examination	0.125		
MT concurrent with benign nodules (+ vs -)	**0.024**	2.078(1.051-4.109)	**0.035**

HR, hazard ratio; CI, confidence interval.

## DISCUSSION

It is generally believed that considerable numbers of patients with low risk thyroid cancer are exposed to the risk of significant side effects and unnecessary surgeries from the current surgical strategy, and screening out patients who do not require immediate surgery is a growing trend in the field of thyroid research. For instance, thyroid tumors diagnosed as the noninvasive encapsulated follicular variant of PTC are not currently defined as cancer [13]. For patients with PTMC, the premise of active surveillance implementation is that this management technique will not affect patients’ quality of life or delay treatment. We all thought establishment of Kuma criteria was a significant try in treatment of PTMC, but what could not be neglected, their conclusions were drawn from auxiliary examination results rather than postoperative data. Because of the limitation of ultrasound, we thought the conclusions lacked certain accuracy. Therefore, in the present study, we expected that information obtained directly from postoperative material could help to identify the indications for operation or surveillance.

Based on the above results, we determined that 80% of patients with PTMC would be considered to have harmless PTMC when adopting the Kuma Hospital screening criteria and that only 15% met the CATO screening criteria. Both criteria showed certain significance for screening harmless PTMC. Some disturbing pathological features of the patients satisfying surveillance conditions formulated by Kuma Hospital decreased significantly indeed. However, the proportion of these features still seemed high, especially CLNM (30.9%), which is not entirely consistent with the study at Kuma Hospital [14]. This also made us realize the limitations of preoperative examination in revealing accurate clinicopathological features. Such a high proportion of patients with pathological risk factors seemed to make them unsuitable for surveillance [15–17]. Moreover, the CATO screening criteria indicated more pronounced effects in identifying harmless PTMC with significantly fewer pathological risk factors, a lower progression rate, and longer DFS. The results shown in Table 3 and Figure 2B and 2C indicate that the Kuma screening criteria actually lacked validity for a proportion of patients in the comparison of the CATO low-risk group and Kuma-CATO group. Furthermore, the strict inclusion conditions for the CATO screening criteria increased sensitivity but meant fewer eligible patients could be enrolled in the group (13.5% in CATO low-risk PTMC group vs. 72.3% in Kuma low-risk PTMC group). Therefore, which kind of strategy should be based on when we choose the conditions of surveillance for patients with PTMC?

Although both criteria cover nodal or distant metastasis, extrathyroidal extension, histology subtype, and tumor location, the CATO screening criteria also include the tumor size, history of radiation exposure, and familial history in addition. We attempted to analyze whether these factors affect the prognosis of PTMC (Tables 4 and 5).

Our results suggest that a familial history is not associated with the prognosis of PTMC because fewer than 40 patients were included, limiting the ability to assess the association between a familial history and recurrence. Previous studies have suggested that second-generation patients with familial nonmedullary thyroid carcinoma exhibited an earlier age of onset and more aggressive clinical characteristics [18, 19]. Additionally, whether patients with PTC with one or two other affected family members can be regarded as having familial nonmedullary thyroid carcinoma is controversial. Mazeh *et al.* [20] found that patients with PTC who had a familial history had more aggressive disease regardless of the number of affected family members.

Tumor size was the most obvious distinguishing condition. Only the CATO screening criteria limited the size of the tumor to ≤5 mm. Previous studies have demonstrated that a tumor diameter of >5 mm was a risk factor for CLNM [21–23]. Lombardi *et al.* [22] also found that a tumor size of >5 mm was related to extracapsular spread. Our study results are similar to these conclusions regarding CLNM. However, the tumor sizes in our study were measured by ultrasound and computed tomography, and the difference in measurements between imaging and pathology must be considered. However, 5 mm as measured by examination certainly could be an appropriate threshold for treatment with surveillance. In addition, Moon *et al.* [24] found that only 1.2% of thyroid malignant nodules measuring ≤5 mm on ultrasonography increased to >3 mm within 12 months, indicating that PTMC lesions of ≤5 mm were less likely to develop. Their study also supports our findings. We therefore propose that redefining PTMC as PTC of ≤5 mm might contribute to management by reasonable surveillance.

Radiation exposure seemed to be a risk factor for disease progression in the survival analysis using the Kaplan–Meier method. Some other studies have also revealed the dangers of radiation exposure in the development of thyroid cancer [25, 26]. Most of these studies were based on the influences of nuclear pollution incidents; however, common radiation exposure incidents in daily life, such as radiotherapy and radioscopy, differ from nuclear pollution incidents in terms of dose, exposure time, and other factors. Few patients in our study had a history of radiation exposure, limiting the accuracy of the results; whether radiation in daily life affects the disease course is unknown based on the present study.

An interesting finding of the current study is that the malignant tumors with concurrent benign nodules seemed to be less invasive than solitary malignant nodules because of the longer DFS in the Cox proportional hazards regression model and less CLNM in the logistic analysis. These patients seem to be more appropriate for surveillance. Whether this phenomenon is caused by the different tumorigenesis of PTMC would be a clinically valuable study topic.

In conclusion, the key to determining the appropriate indications for surveillance is screening out patients with harmless PTMC. When surgeons try to adopt surveillance in patients with tumors, they tend to adopt a conservative, safe way of testing this change. Patients with PTMC exhibiting pathological risk characteristics (CLNM, extrathyroidal extensions, and multifocal lesions) may be more likely to later experience extended surgery or distant metastasis if surgical treatment is not immediately performed. Therefore, the purpose of this study was to identify the criteria that are suitable for subsequent trials. Considering the results of our study, we anticipate that a relatively large proportion of Chinese patients with PTMC will be defined as having harmless cancer when adopting the Kuma Hospital screening criteria, and patients classified in the CATO low-risk criteria will have a lower proportion of clinicopathological risk factors than those classified in the Kuma low-risk criteria. More research is required to determine whether tumors with concurrent benign nodules are more stable for surveillance and whether other prognostic factors are necessary. We also suggest the implementation of a multicenter study to more fully assess the surveillance indications.

## MATERIALS AND METHODS

### Patients

Patients with PTMC who underwent primary operative therapy at Fudan University Shanghai Cancer Center from 2007 to 2010 were enrolled in this retrospective study. All patients included in the study met the following conditions: underwent systematic preoperative testing, had a ≤10-mm maximum diameter of malignant nodules on preoperative ultrasound examination, had no distant metastasis during the initial treatment, had no known history of treatment for thyroid or parathyroid disease before surgery, had follow-up time that was more than 36 months after surgery. Patients with malignant tumors unexpectedly discovered during or after the thyroidectomy were also excluded considering the aim of this study.

### Preoperative tests, surgery and postoperative treatment

Each patient underwent an ultrasonic examination, neck contrast-enhanced CT, and chest X-ray examination before surgery to evaluate the primary lesions and lymph nodes/distant metastasis. Cervical lymph node FNA was carried out if necessary. Thyroid nodule diagnostic FNA was not routinely performed.

Thyroid lobectomy plus ipsilateral central-compartment neck dissection was typically performed in patients with PTMC with malignant lesions confined to a single lobe. Subtotal resection of the contralateral lobe was performed when an obvious benign nodule or undetermined nodule was detected on the other side, and complementary resection was performed if the diagnosis was malignant by intraoperative frozen section. When malignant lesions were found in both lobes of the thyroid or extensive capsular invasion was present even if the lesion was unilateral, total thyroidectomy plus bilateral central-compartment neck dissection was performed. Therapeutic lateral neck compartmental lymph node dissection was performed only for patients with metastatic lateral cervical lymphadenopathy that was either biopsy-proven or highly suspected on imaging. The histological findings of the intraoperative frozen section guided the extent of the surgical procedures in all patients.

For patients who underwent total thyroidectomy, the serum calcium and intact parathyroid hormone concentrations were routinely measured the first day after surgery. These measurements were also performed in patients who underwent lobectomy and showed symptoms of calcium deficiency.

Radioactive iodine remnant ablation was not routinely recommended after thyroidectomy for our patients with PTMC; whether it was necessary was dependent upon the nuclear medicine physicians. All patients received thyroid-stimulating hormone-suppressive therapy after surgery according to the American Thyroid Association guideline. Routine postsurgical examinations including ultrasonic examination, CT, thyroid function testing. FNA and post-treatment whole-body scanning (WBS) or positron emission tomography (PET) were performed during follow-up if indicated.

### Study design

According to the study of Kuma Hospital [11], the following characteristics are absent in patients diagnosed with harmless PTMC: aggressive features such as nodal or distant metastasis, macroscopic extrathyroidal extension, high-grade malignancy on cytology, evidence of progression, and attachment to the trachea or localization along the course of the recurrent laryngeal nerve. Patients with low-risk PTMC as defined by the CATO [12], for whom immediate surgery is not required, should satisfy the following conditions: nonaggressive histology, lesion diameter of ≤5 mm, lesions confined to the gland and no tumor invasion of locoregional tissues or structures, no local or distant metastases, no history of familial thyroid carcinoma history, no history of radiation exposure during childhood or adolescence, no intense mental stress, and active cooperation with the treatment (Table 6). Accordingly, patients who were screened out were divided into low-risk PTMC group defined by Kuma Hospital, high-risk PTMC group defined by Kuma Hospital and low-risk PTMC group defined by CATO, high-risk PTMC group defined by CATO (without considering subjective choices, mental factors, etc.).

**Table 6:** Criteria for PTMC management of active surveillance

Criteria for PTMC management of active surveillance	
Low-risk PTMC conditions defined by Kuma hospital	CATO consensus on PTMC management of active surveillance
No nodal or distant metastasis	Nonaggressive histology
No macroscopic extrathyroidal extension	Diameter≤5mm
No high-grade malignancy on cytology	No familial thyroid carcinoma history
No evidence of progression	No local or distant metastases
No worrisome features (e.g. tumors attached to the trachea or located on the course of the recurrent laryngeal nerve)	Lesions confined to the gland and no tumor invasion of loco-regional tissues or structures
	No history of radiation exposure during the period of teenage or childhood

Treatment outcomes such as the disease progression rate, DFS, clinicopathological characteristics (tumor size, multifocality, extrathyroidal invasion, lymph node metastasis), and surgical complications were compared between the groups. The prognostic indicators in patients with low-risk PTMC were analyzed with the demographic data (age and sex), medical history, and preoperative examination statistics. All patients provided written informed consent, and this study was approved by the Institutional Ethics Committee of Fudan University Shanghai Cancer Center.

### Statistical analyses

The chi-square test or Fisher’s exact probabilities test was used to compare the clinicopathological characteristics of patients between the different groups. The DFS rate was calculated using the Kaplan–Meier method, and groups were compared using the log-rank test. Statistical analyses were performed using logistic regression analysis to evaluate the predictors of CLNM in patients with PTMC. A Cox proportional hazards regression model was used to assess the predictors of DFS. A P value of <0.05 was considered statistically significant. All data obtained in the study were qualitatively and quantitatively analyzed using SPSS 22.0 (IBM Corp., Armonk, NY).

## References

[1] Sobin LH (1990). Histological typing of thyroid tumours. Histopathology.

[2] Vaccarella S, Dal Maso L, Laversanne M, Bray F, Plummer M, Franceschi S (2015). The impact of diagnostic changes on the rise in thyroid cancer incidence: a population-based study in selected high-resource countries. Thyroid.

[3] Vaccarella S, Franceschi S, Bray F, Wild CP, Plummer M, Dal Maso L (2016). Worldwide thyroid-cancer epidemic? The increasing impact of overdiagnosis. N Engl J Med.

[4] Morris LG, Sikora AG, Tosteson TD, Davies L (2013). The increasing incidence of thyroid cancer: the influence of access to care. Thyroid.

[5] Cramer JD, Fu P, Harth KC, Margevicius S, Wilhelm SM (2010). Analysis of the rising incidence of thyroid cancer using the Surveillance, Epidemiology, End Results national cancer data registry. Surgery.

[6] Kim SK, Park I, Woo JW, Lee JH, Choe JH, Kim JH, Kim JS (2016). Predictive factors for lymph node metastasis in papillary thyroid microcarcinoma. Ann Surg Oncol.

[7] Zhang L, Wei WJ, Ji QH, Zhu YX, Wang ZY, Wang Y, Huang CP, Shen Q, Li DS, Wu Y (2012). Risk factors for neck nodal metastasis in papillary thyroid microcarcinoma: a study of 1066 patients. J Clin Endocrinol Metab.

[8] Haugen BR, Alexander EK, Bible KC, Doherty GM, Mandel SJ, Nikiforov YE, Pacini F, Randolph GW, Sawka AM, Schlumberger M, Schuff KG, Sherman SI, Sosa JA (2016). 2015 American Thyroid Association Management Guidelines for adult patients with thyroid nodules and differentiated thyroid cancer: The American Thyroid Association Guidelines Task Force on thyroid nodules and differentiated thyroid cancer. Thyroid.

[9] Brito JP, Hay ID, Morris JC (2014). Low risk papillary thyroid cancer. BMJ.

[10] Brito JP, Ito Y, Miyauchi A, Tuttle RM (2016). A clinical framework to facilitate risk stratification when considering an active surveillance alternative to immediate biopsy and surgery in papillary microcarcinoma. Thyroid.

[11] Oda H, Miyauchi A, Ito Y, Yoshioka K, Nakayama A, Sasai H, Masuoka H, Yabuta T, Fukushima M, Higashiyama T, Kihara M, Kobayashi K, Miya A (2016). Incidences of unfavorable events in the management of low-risk papillary microcarcinoma of the thyroid by active surveillance versus immediate surgery. Thyroid.

[12] Gao M, Ge MH, JI QH, Xu ZG, Lu HK, Cheng RC, Guan HX (2016). Chinese expert consensus on diagnosis and treatment of papillary thyroid microcarcinoma (2016). Chin J Clin Oncol.

[13] Nikiforov YE, Seethala RR, Tallini G, Baloch ZW, Basolo F, Thompson LD, Barletta JA, Wenig BM, Al GA, Kakudo K, Giordano TJ, Alves VA, Khanafshar E (2016). Nomenclature revision for encapsulated follicular variant of papillary thyroid carcinoma: a paradigm shift to reduce overtreatment of indolent tumors. JAMA Oncol.

[14] Ito Y, Miyauchi A, Kihara M, Higashiyama T, Kobayashi K, Miya A (2014). Patient age is significantly related to the progression of papillary microcarcinoma of the thyroid under observation. Thyroid.

[15] Lombardi CP, Bellantone R, De Crea C, Paladino NC, Fadda G, Salvatori M, Raffaelli M (2010). Papillary thyroid microcarcinoma: extrathyroidal extension, lymph node metastases, and risk factors for recurrence in a high prevalence of goiter area. World J Surg.

[16] Pyo JS, Sohn JH, Kang G (2016). Detection of tumor multifocality is important for prediction of tumor recurrence in papillary thyroid microcarcinoma: a retrospective study and meta-analysis. J Pathol Transl Med.

[17] Liu FH, Kuo SF, Hsueh C, Chao TC, Lin JD (2015). Postoperative recurrence of papillary thyroid carcinoma with lymph node metastasis. J Surg Oncol.

[18] Capezzone M, Marchisotta S, Cantara S, Busonero G, Brilli L, Pazaitou-Panayiotou K, Carli AF, Caruso G, Toti P, Capitani S, Pammolli A, Pacini F (2008). Familial non-medullary thyroid carcinoma displays the features of clinical anticipation suggestive of a distinct biological entity. Endocr Relat Cancer.

[19] Park YJ, Ahn HY, Choi HS, Kim KW, Park DJ, Cho BY (2012). The long-term outcomes of the second generation of familial nonmedullary thyroid carcinoma are more aggressive than sporadic cases. Thyroid.

[20] Mazeh H, Benavidez J, Poehls JL, Youngwirth L, Chen H, Sippel RS (2012). In patients with thyroid cancer of follicular cell origin, a family history of nonmedullary thyroid cancer in one first-degree relative is associated with more aggressive disease. Thyroid.

[21] So YK, Son YI, Hong SD, Seo MY, Baek CH, Jeong HS, Chung MK (2010). Subclinical lymph node metastasis in papillary thyroid microcarcinoma: a study of 551 resections. Surgery.

[22] Lombardi CP, Bellantone R, De Crea C, Paladino NC, Fadda G, Salvatori M, Raffaelli M (2010). Papillary thyroid microcarcinoma: extrathyroidal extension, lymph node metastases, and risk factors for recurrence in a high prevalence of goiter area. World J Surg.

[23] Zhang L, Yang J, Sun Q, Liu Y, Liang F, Liu Z, Chen G, Chen S, Shang Z, Li Y, Li X (2016). Risk factors for lymph node metastasis in papillary thyroid microcarcinoma: Older patients with fewer lymph node metastases. Eur J Surg Oncol.

[24] Moon HJ, Lee HS, Kim EK, Ko SY, Seo JY, Park WJ, Park HY, Kwak JY (2015). Thyroid nodules ≤ 5 mm on ultrasonography: are they "leave me alone" lesions?. Endocrine.

[25] Hatch M, Brenner A, Bogdanova T, Derevyanko A, Kuptsova N, Likhtarev I, Bouville A, Tereshchenko V, Kovgan L, Shpak V, Ostroumova E, Greenebaum E, Zablotska L (2009). A screening study of thyroid cancer and other thyroid diseases among individuals exposed in utero to iodine-131 from Chernobyl fallout. J Clin Endocrinol Metab.

[26] Michel LA, Donckier J, Rosiere A, Fervaille C, Lemaire J, Bertrand C (2016). Post-Chernobyl incidence of papillary thyroid cancer among Belgian children less than 15 years of age in April 1986: a 30-year surgical experience. Acta Chir Belg.

